# ATP Mediates NADPH Oxidase/ROS Generation and COX-2/PGE_2_ Expression in A549 Cells: Role of P2 Receptor-Dependent STAT3 Activation

This article has been retracted.

**DOI:** 10.1371/journal.pone.0054125

**Published:** 2013-01-11

**Authors:** Shin-Ei Cheng, I-Ta Lee, Chih-Chung Lin, Wan-Ling Wu, Li-Der Hsiao, Chuen-Mao Yang

**Affiliations:** 1 Department of Physiology and Pharmacology and Health Aging Research Center, College of Medicine, Chang Gung University, Kwei-San, Tao-Yuan, Taiwan; 2 Department of Anesthetics, Chang Gung Memorial Hospital at Lin-Kou and College of Medicine, Chang Gung University, Kwei-San, Tao-Yuan, Taiwan; National Cancer Institute (INCA), Brazil

## Abstract

**Background:**

Up-regulation of cyclooxygenase (COX)-2 and its metabolite prostaglandin E_2_ (PGE_2_) are frequently implicated in lung inflammation. Extracellular nucleotides, such as ATP have been shown to act via activation of P2 purinoceptors, leading to COX-2 expression in various inflammatory diseases, such as lung inflammation. However, the mechanisms underlying ATP-induced COX-2 expression and PGE_2_ release remain unclear.

**Principal Findings:**

Here, we showed that ATPγS induced COX-2 expression in A549 cells revealed by western blot and real-time PCR. Pretreatment with the inhibitors of P2 receptor (PPADS and suramin), PKC (Gö6983, Gö6976, Ro318220, and Rottlerin), ROS (Edaravone), NADPH oxidase [diphenyleneiodonium chloride (DPI) and apocynin], Jak2 (AG490), and STAT3 [cucurbitacin E (CBE)] and transfection with siRNAs of PKCα, PKCι, PKCμ, p47*^phox^*, Jak2, STAT3, and cPLA_2_ markedly reduced ATPγS-induced COX-2 expression and PGE_2_ production. In addition, pretreatment with the inhibitors of P2 receptor attenuated PKCs translocation from the cytosol to the membrane in response to ATPγS. Moreover, ATPγS-induced ROS generation and p47*^phox^* translocation was also reduced by pretreatment with the inhibitors of P2 receptor, PKC, and NADPH oxidase. On the other hand, ATPγS stimulated Jak2 and STAT3 activation which were inhibited by pretreatment with PPADS, suramin, Gö6983, Gö6976, Ro318220, GF109203X, Rottlerin, Edaravone, DPI, and apocynin in A549 cells.

**Significance:**

Taken together, these results showed that ATPγS induced COX-2 expression and PGE_2_ production via a P2 receptor/PKC/NADPH oxidase/ROS/Jak2/STAT3/cPLA_2_ signaling pathway in A549 cells. Increased understanding of signal transduction mechanisms underlying COX-2 gene regulation will create opportunities for the development of anti-inflammation therapeutic strategies.

## Introduction

Lung inflammation is a pivotal event in the pathogenesis of chronic obstructive pulmonary disease and asthma [1]. Cyclooxygenases (COXs) are responsible for the formation of prostaglandins (PGs), which are involved in inflammatory responses [2]. COX-2 is primarily an inducible isoform whose expression can be up-regulated by cytokines, mitogens, and endotoxins in many cell types [2]. It is highly expressed in inflamed tissues and believed to produce PGs involved in inflammatory processes [3]. Moreover, the physiological relevance of the purinergic signaling network for airway defenses is emerging through cumulating reports of abnormal ATP and adenosine levels in the airway secretions of patients with asthma and chronic pulmonary obstructive diseases. The consequences for airway defenses range from abnormal clearance responses to the destruction of lung tissue by inflammation [4]. Thus, to clarify the mechanisms of COX-2 induction by ATP in lung epithelium was recognized as a new therapeutic approach in the management of respiratory diseases.

ATP transports chemical energy within cells, is produced by cellular respiration and is used by enzymes and structural proteins in many cellular processes [5]. Extracellular ATP is an important mediator of intercellular communication via the activation of purinergic P2X and P2Y receptors mediated through ion channels and GTP binding protein coupled receptors, respectively [6]. Growing evidence indicates the involvement of ATP and purinoceptors in the pathogenesis of lung diseases [5], [6]. ATP has been shown to induce COX-2 expression [7], [8], and then causes the inflammatory responses. However, the mechanisms by which ATP induced COX-2 expression in A549 cells are not completely understood.

Oxidative stress is an important factor in the pathogenesis of respiratory diseases. Excessive ROS can directly damage cellular macromolecules, resulting in cell cycle arrest and/or cell death [9]. NADPH oxidase is an enzymatic source for the production of ROS under various pathologic conditions [10]. Activated NADPH oxidase is a multimeric protein complex consisting of at least three cytosolic subunits of p47*^phox^*, p67*^phox^*, and p40*^phox^*. The p47*^phox^* regulatory subunit plays a critical role in acute activation of NADPH oxidase; phosphorylation of p47*^phox^* is thought to relieve inhibitory intracellular interactions and permit the binding of p47*^phox^* to p22*^phox^*, thereby increasing NADPH oxidase activation [10]. ROS have been shown to regulate COX-2 expression and induce inflammation [11]. In addition, protein kinase C (PKC) has been involved in the transduction of signals for cell proliferation and differentiation [12]. Some studies have indicated that the expression of COX-2 is mediated by the activation of PKC [13], [14]. PKC has also been shown to stimulate NADPH oxidase activity and ROS generation [15]. Here, we investigated the role of PKC in ATP-induced ROS generation and COX-2 expression.

Signal transducer and activator of transcription (STAT)3 belongs to the STAT family. STAT3 was first identified and cloned from mouse liver cDNA library in the study of IL-6 signaling [16]. Like its relatives, STAT3 is inactive in nonstimulated cells, but is rapidly activated by various cytokines and growth factors [16]. The phosphorylation of STAT3 at Tyr^705^ is most commonly mediated by Janus kinases (Jaks), especially Jak2 [17]. COX-2 expression has also been shown to be mediated via Jak2/STAT3 activation in various cell types [18], [19]. These findings imply that these signaling components Jak2/STAT3 might be also implicated in the expression of COX-2 induced by ATP in A549 cells.

Therefore, ATP may play a potential role in regulation of expression of inflammatory genes, such as COX-2 and thereby promote inflammatory responses. We report here for the first time that ATPγS-induced COX-2 expression was mediated through a P2 receptor/PKC/NADPH oxidase/ROS/Jak2/STAT3-dependent pathway in A549 cells.

## Methods

### Materials

Anti-cPLA_2_, anti-PKCα, anti-PKCι, anti-PKCμ, anti-STAT3, anti-Jak2, anti-β-actin, and anti-p47*^phox^* antibodies were from Santa Cruz (Santa Cruz, CA). Anti-COX-2 antibody was from BD Transduction Laboratories (San Diego, CA). Adenosine 5′-O-(3-thiotriphosphate) (ATPγS), Gö6983, Gö6976, GF109203X, Ro318220, Rottlerin, PPADS, suramin, AG490, CBE, and arachidonic acid were from Biomol (Plymouth Meeting, PA). All other chemicals and enzymes were obtained from Sigma (St. Louis, MO). Edaravone (MCI-186) was from Tocris Bioscience (Ellisville, MO). CellROX™ Deep Red Reagent and CM-H_2_DCFDA were from Invitrogen (Carlsbad, CA).

### Cell Culture

A549 cells (human alveolar epithelial cell carcinoma) were purchased from the American Type Culture Collection (Manassas, VA) and grown as previously described [20].

### Western Blot Analysis

Growth-arrested A549 cells were incubated with ATPγS at 37°C for the indicated time intervals. The cells were washed, scraped, collected, and centrifuged at 45000×*g* at 4°C for 1 h to yield the whole cell extract, as previously described [20]. Samples were denatured, subjected to SDS-PAGE using a 12% running gel, transferred to nitrocellulose membrane, incubated with an anti-COX-2 or anti-cPLA_2_ antibody for 24 h, and then incubated with an anti-mouse horseradish peroxidase Ab for 1 h. The immunoreactive bands were detected by ECL reagents and analyzed by using a UN-SCAN-IT Gel 6.1 program (Silk Scientific, Inc., Orem, UT).

### Real-time PCR

Total RNA was extracted using TRIzol reagent. mRNA was reverse-transcribed into cDNA and analyzed by real-time RT-PCR. Real-time PCR was performed using SYBR Green PCR reagents (Applied Biosystems, Branchburg, NJ) and primers specific for COX-2 and GAPDH mRNAs. The levels of COX-2 expression were determined by normalizing to GAPDH expression.

### Isolation of Cell Fractions

Cells were harvested, sonicated for 5 s at output 1.5 with a sonicator (Misonix Inc., Farmingdale, NY), and centrifuged at 8000 rpm for 15 min at 4°C. The pellet was collected as the nuclear fraction. The supernatant was centrifuged at 14000 rpm for 60 min at 4°C to yield the pellet (membrane fraction) and the supernatant (cytosolic fraction).

### Determination of NADPH Oxidase Activity by Chemiluminescence Assay

Cells grew onto 6-well culture plates, after exposure to ATPγS for the indicated time intervals, were gently scraped and centrifuged at 400×*g* for 10 min at 4°C. The cell pellet was re-suspended in 35 µl/per vial of ice-cold RPMI-1640 medium (Gibco BRL, Grand Island, NY), and the cell suspension was kept on ice. To a final 200 µl volume of pre-warmed (37°C) RPMI-1640 medium containing either NADPH (1 µM) or lucigenin (20 µM), 5 µl of cell suspension (0.2×10^5^ cells) was added to initiate the reaction followed by immediate measurement of chemiluminescence in an Appliskan luminometer (Thermo®) in out-of-coincidence mode. Appropriate blanks and controls were established, and chemiluminescence was recorded. Neither NADPH nor NADH enhanced the background chemiluminescence of lucigenin alone (30−40 counts per min). Chemiluminescence was measured continuously for 12 min, and the activity of NADPH oxidase was expressed as counts per million cells.

### Measurement of Intracellular ROS Accumulation

The intracellular H_2_O_2_ levels were determined by measuring fluorescence of DCF-DA. A549 cells were washed with warm HBSS and incubated in HBSS containing 10 µM DCFH-DA at 37°C for 45 min. Subsequently, HBSS containing DCFH-DA was removed and replaced with fresh cell medium. Cells were then incubated with various concentrations of ATPγS. Cells were washed twice with PBS and detached with trypsin/EDTA, and the fluorescence intensity of the cells was analyzed using a FACScan flow cytometer (BD Biosciences, San Jose, CA) at 495-nm excitation and 529-nm emission for DCF. In addition, CellROX™ Deep Red Reagent is a fluorogenic probe designed to reliably measure ROS in living cells. The cell-permeable CellROX™ Deep Red dye is nonfluorescent while in a reduced state and upon oxidation exhibits excitation/emission maxima at 640/665 nm. A549 cells were treated with ATPγS for the indicated time intervals, CellROX™ Deep Red Reagent was added at a final concentration of 5 µM to the cells, and then incubated for 30 min at 37°C. Subsequently, medium was removed and the cells were washed three times with PBS. The resulting fluorescence was measured using a fluorescence microscope (Zeiss, Axiovert 200M).

### Transient Transfection with siRNAs

The small interfering RNA (siRNA) duplexes corresponding to human cPLA_2_, PKCα, PKCι, PKCμ, p47*^phox^*, Jak2, and STAT3 and scrambled siRNA were from Invitrogen (Carlsbad, CA). Transient transfection of siRNAs was carried out using Metafectene transfection reagent. siRNA (100 nM) was formulated with Metafectene transfection reagent according to the manufacturer’s instruction (Biontex Lab. GmbH, Planegg/Martinsried, Germany).

### Measurement of PGE_2_ Generation

A549 cells were cultured in 6-well culture plates. After reaching confluence, growth-arrested cells were treated with ATPγS for the indicated time intervals at 37°C. The medium were collected and stored at −80°C until being assayed. PGE_2_ was assayed using a PGE_2_ enzyme immunoassay kit (Cayman) according to the manufacturer’s instructions.

### Analysis of Data

All the data were estimated using the GraphPad Prism Program (GraphPad, San Diego, CA). Data were expressed as the mean±SEM and analyzed with a one-way ANOVA followed with Tukey’s post-hoc test at *p*<0.05 level of significance. All the experiments were performed at least three times.

## Results

### ATPγS Induces COX-2 Expression via a PKCs Signaling

PKCs have been shown to be involved in proliferation and differentiation [12]. Some studies have indicated that the expression of COX-2 is mediated by the activation of PKCs [13], [14]. Here, we investigated the role of PKCs in ATPγS-induced COX-2 expression. As shown in Fig. 1A, pretreatment with the inhibitor of non-selective PKC (Ro318220), Ca^2+^-dependent PKC (Gö6983 and Gö6976), or selective PKCδ (Rottlerin) markedly attenuated ATPγS-induced COX-2 expression in A549 cells. COX-2 is the enzyme which converts arachidonic acid to PGH_2_, which can be further metabolized to prostanoids, including PGE_2_, prostacyclin (PGI_2_), and thromboxane A_2_ (TXA_2_) [21]. Pretreatment with these inhibitors also attenuated ATPγS-induced COX-2 mRNA expression and PGE_2_ generation (Fig. 1B). Translocation of PKC from the cytosol to the membrane is necessary to activation of PKC [12]. Next, we investigated whether ATPγS could stimulate PKCs translocation in A549 cells. As shown in Fig. 1C, ATPγS and PMA (a PKCs activator) stimulated the translocation PKCα, PKCι, and PKCμ from the cytosol to the membrane in a time-dependent manner. Moreover, to further ascertain the role of PKCs in ATPγS-induced COX-2 protein expression, as shown in Figs. 1D and E, transfection with siRNAs of PKCα, PKCι, and PKCμ down-regulated PKCα, PKCι, and PKCμ protein expression, respectively, and then reduced ATPγS-induced COX-2 expression and PGE_2_ production. These data demonstrated that PKCs play an important role in ATPγS-induced COX-2 expression in A549 cells.

**Figure 1:** ATPγS regulates COX-2 expression via PKCs in A549 cells. Cells were pretreated with Gö6983, Gö6976, Ro318220, or Rottlerin for 1 h, and then incubated with ATPγS for (A) 6 h or (B) 2 h. The levels of COX-2 (A) protein and (B) mRNA were analyzed by western blot and real-time PCR, respectively. (A) The media were collected and analyzed for PGE_2_ release. (C) Cells were treated with ATPγS (100 µM) for the indicated time intervals or PMA (1 µM) for 15 min. The cytosolic and membrane fractions were prepared and analyzed by western blot using an anti-PKCα, anti-PKCι, or anti-PKCμ antibody. β-actin and Gαs were used as a marker protein for cytosolic and membrane fractions, respectively. (D, E) Cells were transfected with siRNA of scrambled, PKCα, PKCι, or PKCμ, and then incubated with ATPγS for 6 h. The expression of PKCα, PKCι, PKCμ, and COX-2 were analyzed by western blot. The media were collected and analyzed for PGE_2_ release. Data are expressed as mean±S.E.M. of three independent experiments. *p<0.5; ^#^ *p*<0.01, as compared with the cells exposed to ATPγS alone (A, B) or the cells transfected with scrambled siRNA and exposed to ATPγS alone (D, E).

### NADPH Oxidase/ROS are Involved in ATPγS-induced COX-2 Expression

NADPH oxidase is an enzymatic source for the production of ROS under various pathological conditions [11]. ROS has been shown to induce COX-2 expression associated with inflammation [11]. Thus, the role of NADPH oxidase/ROS generation in ATPγS-induced COX-2 expression was investigated. As shown in Fig. 2A, pretreatment of A549 cells with NADPH oxidase inhibitors [DPI and apocynin (APO)] or a ROS inhibitor (Edaravone) significantly abrogated ATPγS-induced COX-2 protein expression. In addition, pretreatment with these inhibitors also attenuated ATPγS-induced COX-2 mRNA expression and PGE_2_ generation (Fig. 2B). To further ascertain that generation of ROS was involved in ATPγS-induced COX-2 expression, a fluorescent probe, DCFH-DA, was used to determine the generation of ROS in A549 cells. As illustrated in Figs. 2C and D, ATPγS induced a significant increase in NADPH oxidase activity and ROS generation within 15 min, reached a peak within 60 min, and slightly declined within 120 min. Pretreatment with Eadaravone, DPI, and APO attenuated ATPγS-induced NADPH oxidase/ROS generation. On the other hand, we used CellROX™ Deep Red Reagent to confirm the generation of ROS in ATPγS-stimulated A549 cells. As shown in Figs. 2E and F, ATPγS induced ROS generation in a time-dependent manner, which was also attenuated by pretreatment with Edaravone, DPI, or APO in these cells. Activated NADPH oxidase is a multimeric protein complex consisting of at least three cytosolic subunits of p47*^phox^*, p67*^phox^*, and p40*^phox^*. It has been demonstrated that p47*^phox^* organizes the translocation of other cytosolic factors, hence its designation as “organizer subunit” [22]. Here, we found that ATPγS induced a significant translocation of p47*^phox^* from the cytosol to the membrane (Fig. 2G). The role of p47*^phox^* in ATPγS-mediated responses was also confirmed by transfection with p47*^phox^* siRNA which down-regulated p47*^phox^* protein expression, and then attenuated COX-2 expression and PGE_2_ production induced by ATPγS in A549 cells (Figs. 2H and I). These results indicated that NADPH oxidase activation and ROS generation play critical roles in ATPγS-induced COX-2 expression in A549 cells.

**Figure 2:** ATPγS induces NADPH oxidase-dependent COX-2 expression in A549 cells. Cells were pretreated with Edaravone, DPI, or APO for 1 h, and then incubated with ATPγS for (A) 6 h or (B) 2 h. The levels of COX-2 (A) protein and (B) mRNA were analyzed by western blot and real-time PCR, respectively. (A) The media were collected and analyzed for PGE_2_ release. Cells were labeled with DCF-DA (10 µM), and then incubated with ATPγS (100 µM) for (C) the indicated time intervals or (D) pretreated with Edaravone (10 µM), DPI (10 µM), or APO (100 µM) for 1 h, and then stimulated with ATPγS (100 µM) for 1 h. The fluorescence intensity (relative DCF fluorescence) was measured and NADPH oxidase activity was determined. Cells were treated with (E) ATPγS for the indicated time intervals or (F) pretreated with Edaravone (10 µM), DPI (10 µM), or APO (100 µM) for 1 h, and then stimulated with ATPγS (100 µM) for 1 h. After incubation, CellROX™ Deep Red Reagent was added at a final concentration of 5 µM to the cells, and then incubated for 30 min at 37°C. Subsequently, medium was removed and the cells were washed thrice with PBS. The resulting fluorescence was measured using a fluorescence microscope. (G) Cells were incubated with ATPγS (100 µM) for the indicated time intervals. The membrane and cytosolic fractions were prepared and analyzed by western blot using an anti-p47*^phox^* antibody. (H, I) Cells were transfected with siRNA of scrambled or p47*^phox^*, and then incubated with ATPγS for 6 h. The levels of p47*^phox^* and COX-2 expression were analyzed by western blot. The media was collected and analyzed for PGE_2_ release. Data are expressed as mean±S.E.M. of three independent experiments. *p<0.5; ^#^ *p*<0.01, as compared with the cells exposed to ATPγS alone (A, B, D), the cells exposed to vehicle alone (C), or the cells transfected with scrambled siRNA and exposed to ATPγS alone (H, I).

### ATPγS Induces NADPH Oxidase Activation and ROS Production via PKCs

PKCs have also been shown to stimulate NADPH oxidase activity and ROS generation [15]. Thus, we investigated whether ATPγS stimulated NADPH oxidase activation and ROS production via PKCs activation in A549 cells. As shown in Figs. 3A and B, pretreatment with Ro318220, GF109203X, Gö6983, Gö6976, or Rottlerin markedly inhibited ATPγS-stimulated NADPH oxidase activity and H_2_O_2_ and/or ROS generation. In addition, pretreatment with these inhibitors also reduced p47*^phox^* translocation from the cytosol to the membrane (Fig. 3C). These data suggested that PKC plays a key role in ATPγS-stimulated NADPH oxidase activation and ROS production in A549 cells.

**Figure 3:** ATPγS induces PKC-dependent ROS generation in A549 cells. (A) Cells were labeled with DCF-DA (10 µM), pretreated with Gö6983 (10 µM), Gö6976 (10 µM), GF109203X (3 µM), Ro318220 (10 µM), or Rottlerin (10 µM) for 1 h, and then incubated with ATPγS for 1 h. The fluorescence intensity (relative DCF fluorescence) was measured (gray bar). In addition, NADPH oxidase activity was determined (white bar). (B) Cells were pretreated with Gö6983 (10 µM), Gö6976 (10 µM), GF109203X (3 µM), Ro318220 (10 µM), or Rottlerin (10 µM) for 1 h, and then incubated with ATPγS for 1 h. After incubation, ROS generation was determined by using CellROX™ Deep Red Reagent as described in Fig. 2E. (C) Cells were pretreated with Gö6983 (10 µM), Gö6976 (10 µM), GF109203X (3 µM), Ro318220 (10 µM), or Rottlerin (10 µM) for 1 h, and then incubated with ATPγS for 1 h. The membrane and cytosolic fractions were prepared and analyzed by western blot using an anti-p47*^phox^* antibody. Data are expressed as mean±S.E.M. of three independent experiments. ^#^ *p*<0.01, as compared with the cells exposed to ATPγS alone.

### ATPγS Induces COX-2 Expression via P2 Receptors

Extracellular nucleotides regulate ion transport and inflammatory responses of the lung epithelium by activation of P2 receptors [12]. To investigate whether ATPγS could induce COX-2 expression, PKCs translocation, and ROS generation via P2 receptors, the P2Y and P2X receptor antagonists, suramin and PPADS were used. As shown in Figs. 4A and B, pretreatment with PPADS or suramin markedly inhibited ATPγS-induced COX-2 protein and mRNA expression and PGE_2_ production. ATPγS-stimulated ROS production, NADPH oxidase activity, and p47*^phox^* translocation was also inhibited by pretreatment with PPADS or suramin in A549 cells (Figs. 4C–E). In addition, pretreatment with PPADS or suramin also reduced PKCα, PKCι, and PKCμ translocation from the cytosol to the membrane in response to ATPγS (Fig. 4F). These data demonstrated that ATPγS induces COX-2 expression via P2 receptors in A549 cells.

**Figure 4:** ATPγS induces P2 receptor-dependent COX-2 expression, PKC translocation, and ROS generation in A549 cells. Cells were pretreated with PPADS or suramin for 1 h, and then treated with ATPγS for (A) 6 h or (B) 2 h. The levels of COX-2 (A) protein and (B) mRNA were analyzed by western blot and real-time PCR, respectively. (A) The media were collected and analyzed for PGE_2_ release. (C) Cells were labeled with DCF-DA (10 µM), pretreated with PPADS or suramin for 1 h, and then incubated with ATPγS for 1 h. The fluorescence intensity (relative DCF fluorescence) was measured (gray bar). In addition, NADPH oxidase activity was determined (white bar). (D) Cells were pretreated with PPADS or suramin for 1 h, and then incubated with ATPγS for 1 h. After incubation, ROS generation was determined by using CellROX™ Deep Red Reagent as described in Fig. 2E. (E) Cells were pretreated with PPADS (10 µM) or suramin (10 µM) for 1 h, and then incubated with ATPγS for 1 h. The membrane and cytosolic fractions were prepared and analyzed by western blot using an anti-p47*^phox^* antibody. (F) Cells were pretreated with PPADS (10 µM) or suramin (10 µM) for 1 h, and then treated with ATPγS for 15 min. The cytosolic and membrane fractions were prepared and analyzed by western blot using an anti-PKCα, anti-PKCι, or anti-PKCμ antibody. Data are expressed as mean±S.E.M. of three independent experiments. ^#^ *p*<0.01, as compared with the cells exposed to ATPγS alone.

### Jak2/STAT3 are Involved in ATPγS-induced COX-2 Expression

STAT3 is a transcription factor that is activated by many cytokines and growth factors and plays a key role in cell survival, proliferation, and differentiation [23]. The phosphorylation of STAT3 at Tyr^705^ is most commonly mediated by Jaks, especially Jak2 [17]. Thus, we also evaluated whether Jak2 and STAT3 were involved in ATPγS-induced COX-2 expression in A549 cells. As shown in Figs. 5A and B, pretreatment with the inhibitors of Jak2 (AG490) and STAT3 (CBE) reduced ATPγS-induced COX-2 protein and mRNA expression and PGE_2_ production. Moreover, ATPγS stimulated Jak2 and STAT3 phosphorylation in a time-dependent manner (Fig. 5C). In response to cytokines and growth factors, STAT family members are phosphorylated by receptor-associated kinases and then form homo- or heterodimers that translocate into the nucleus, where they act as transcription activators [23]. Next, we showed that ATPγS markedly induced STAT3 translocation in a time-dependent manner in A549 cells (Fig. 5D), which was inhibited by pretreatment with AG490, CBE, PPADS, and suramin in A549 cells (Fig. 5E). We further confirm the roles of Jak2 and STAT3 in ATPγS-induced responses by using siRNAs of Jak2 and STAT3. Here, we showed that ATPγS-induced COX-2 expression and PGE_2_ generation was reduced by transfection with siRNA of Jak2 or STAT3 (Figs. 5F and G). These results showed that ATPγS induces COX-2 expression via a P2 receptor/Jak2/STAT3 signaling in A549 cells.

**Figure 5:** ATPγS induces COX-2 expression via Jak2/STAT3 in A549 cells. Cells were pretreated with AG490 or CBE for 1 h, and then incubated with ATPγS for (A) 6 h or (B) 2 h. The levels of COX-2 (A) protein and (B) mRNA were analyzed by western blot and real-time PCR, respectively. (A) The media were collected and analyzed for PGE_2_ release. (C) Cells were treated with ATPγS (100 µM) for the indicated time intervals. The cell lysates were analyzed by western blot using an anti-phospho-Jak2, anti-phospho-STAT3, anti-STAT3, or anti-β-actin antibody. Cells were pretreated (D) without or (E) with AG490 (10 µM), CBE (10 µM), PPADS (10 µM), or suramin (10 µM) for 1 h, and then incubated with ATPγS (100 µM) for (D) the indicated time intervals or (E) 60 min. The cytosolic and nuclear fractions were prepared and analyzed by western blot using an anti-phospho-STAT3 or anti-STAT3 antibody. GAPDH and Lamin A were used as a marker protein for cytosolic and nuclear fractions, respectively. (F) Cells were transfected with siRNA of scrambled, Jak2, or STAT3, and then incubated with ATPγS for 6 h. The levels of Jak2, STAT3, and COX-2 expression were analyzed by western blot. The media were collected and analyzed for PGE_2_ release. Data are expressed as mean±S.E.M. of three independent experiments. ^#^ *p*<0.01, as compared with the cells exposed to ATPγS alone (A, B), the cells exposed to vehicle alone (C), or the cells transfected with scrambled siRNA and exposed to ATPγS alone (F, G).

### ATPγS Stimulates Jak2/STAT3 Activation via a PKCs/ROS Signaling

We further investigated whether PKCs and NADPH oxidase/ROS were involved in ATPγS-stimulated Jak2 and STAT3 activation in A549 cells. We found that ATPγS-stimulated Jak2 and STAT3 translocation and phosphorylation was reduced by pretreatment with Edaravone, APO, DPI, Ro318220, GF109203X, Gö6983, Gö6976, or Rottlerin and transfection with siRNAs of p47*^phox^*, PKCα, PKCι, and PKCμ (Figs. 6A and B). These results demonstrated that ATPγS stimulates Jak2 and STAT3 activation via PKC/NADPH oxidase/ROS in A549 cells.

**Figure 6:** ATPγS regulates PKC/ROS-dependent Jak2 and STAT3 activation in A549 cells. (A) Cells were pretreated with APO (100 µM), DPI (10 µM), Edaravone (10 µM), Gö6983 (10 µM), Gö6976 (10 µM), GF109203X (3 µM), Ro318220 (10 µM), or Rottlerin (10 µM) for 1 h, and then incubated with ATPγS for 1 h. The cytosolic and nuclear fractions were prepared and subjected to Western blot analysis using an anti-phospho-STAT3 or anti-STAT3 antibody. (B) Cells were transfected with siRNAs of scrambled, p47*^phox^*, PKCα, PKCι, and PKCμ, and then incubated with ATPγS for 1 h. The cell lysates were subjected to western blot analysis using an anti-phospho-Jak2, anti-phospho-STAT3, or anti-β-actin antibody. Data are expressed as mean±S.E.M. of three independent experiments. ^#^ *p*<0.01, as compared with the cells exposed to scrambled siRNA+ATPγS.

### ATPγS Induces COX-2/PGE_2_ Expression via a cPLA_2_/AA Pathway

Indeed, cytosolic phospholipase A_2_ (cPLA_2_) is also involved in PGE_2_ production. As shown in Fig. 7A, ATPγS markedly induced cPLA_2_ and COX-2 expression in a time-dependent manner in A549 cells. However, ATPγS had no effect on COX-1 expression in A549 cells. We also found that ATPγS-induced COX-2 expression was inhibited by transfection with siRNA of cPLA_2_ or COX-2 (Fig. 7B). Moreover, COX-2 siRNA had no effects on ATPγS-induced cPLA_2_ protein expression (Fig. 7B). These data suggested that ATPγS induced COX-2 expression via a cPLA_2_-dependent pathway. We further found that arachidonic acid (AA) markedly enhanced COX-2, but not COX-1 expression in A549 cells (Fig. 7C). Finally, we observed that AA and ATPγS induced PGE_2_ production (Fig. 7D). Moreover, ATPγs-induced PGE_2_ production was reduced by transfection with siRNA of cPLA_2_ or COX-2 (Fig. 7E). These results suggested that ATPγS induced PGE_2_ production via a cPLA_2_/AA/COX-2 pathway in A549 cells. On the other hand, we found that ATPγS-induced cPLA_2_ expression was reduced by the inhibitors of PKCs, ROS, Jak2, and STAT3 in A549 cells (data not shown). Thus, we suggested that ATPγ induced PGE_2_ production via a P2 receptor/PKC/NADPH oxidase/ROS/Jak2/STAT3/cPLA_2_/AA/COX-2 pathway in A549 cells.

**Figure 7:** ATPγS induces COX-2 expression via a cPLA_2_/AA signaling. (A) Cells were treated with ATPγS for the indicated times. The expression of cPLA_2_, COX-2, or COX-1 was determined by Western blot. (B) Cells were transfected with cPLA_2_ or COX-2 siRNA, and then treated with ATPγS for 24 h or 6 h. The expression of cPLA_2_ or COX-2 was determined by Western blot. (C) Cells were treated with AA for the indicated times. The expression of COX-2 or COX-1 was determined by Western blot. (D) Cells were treated with ATPγS or AA for the indicated times. The production of PGE_2_ was measured. (E) Cells were transfected with cPLA_2_ or COX-2 siRNA, and then treated with ATPγS for 6 h. The production of PGE_2_ was measured. Data are expressed as mean±S.E.M. of three independent experiments. ^#^ *p*<0.01, as compared with the cells exposed to vehicle alone (D) or scrambled siRNA+ATPγS (E).

## Discussion

Asthma and COPD are pulmonary disorders characterized by various degrees of inflammation and tissue remodeling. ATP is a major signaling molecule in the patients with asthma and COPD [4], [5]. ATP elicits its actions by engaging cell surface purinoceptors, and substantial preclinical evidence suggests that targeting these receptors will provide novel approaches for the treatment of asthma and COPD [4], [5]. Patients with COPD show evidence of increased release of ROS leading to oxidative stress [24]. On the other hand, several lines of evidence suggest that high levels of PGs, synthesized by COX-2, are involved in inflammatory responses [25]. The molecular mechanisms by which ATP induces COX-2-dependent PGE_2_ generation are not fully understood in A549 cells. The present study clearly demonstrated that COX-2 expression induced by ATPγS was mediated through a P2 receptor/PKC/NADPH oxidase/Jak2/STAT3/cPLA_2_ pathway. Genetic silencing through transfection with siRNA of cPLA_2_, PKCα, PKCι, PKCμ, p47*^phox^*, Jak2, or STAT3 or pretreatment with the inhibitors of P2 receptors, PKCs, NADPH oxidase, Jak2, and STAT3 abrogated ATPγS-induced COX-2 expression and PGE_2_ release. Therefore, P2 receptor activation by ATPγS causes inflammatory responses through ROS and PGE_2_ production. Moreover, PKC, NADPH oxidase, Jak2, and STAT3 were also involved in ATPγS-induced COX-2 expression in A549 cells (Fig. 7).

Extracellular adenosine 5'-triphosphate (eATP) is ubiquitously used for cell-to-cell communication [5]. The low level of eATP that exists in a “halo” surrounding resting cells signals the presence of neighboring living cells. Larger increases in eATP that are associated with cell death serve as a key “danger” signal in inflammatory processes [26]. Various aspects of purinergic signaling have been demonstrated in different cell types [12], [27], [28]. PKC represents a family of more than 11 phospholipid-dependent Ser/Thr kinases that are involved in a variety of pathways that regulate cell growth, death, and stress responsiveness [29]. PKC isoforms are divided into three categories according to the cofactors that are required for optimal phospholipid-dependent catalytic activity [29]. ATP has been shown to regulate PKC activation [12], [30]. In addition, PKC plays a key role in regulating COX-2 induction [14], [31]. Indeed, we showed that COX-2 expression and PGE_2_ production in response to ATPγS were significantly reduced by transfection with siRNAs of PKCα, PKCι, and PKCμ or pretreatment with the inhibitors of PKCs in A549 cells. Translocation to the membrane is necessary to activate PKC [12]. This notion is confirmed by our observation that ATPγS stimulated PKCs translocation from the cytosol to the membrane. These results suggested that ATPγS plays an important role in PKCs activation leading to COX-2/PGE_2_ expression in A549 cells.

Cells and tissues are routinely subjected to sublethal doses of various oxidants, either exogenously through environmental exposure or endogenously through inflammatory processes [24], [29]. The biological function of NADPH oxidase enzymes might be attributable to the production of ROS [24]. Activation of the NADPH oxidase, *i.e.* activation of gp91*^phox^*, requires stimulus-induced membrane translocation of cytosolic proteins, including the small GTPase Rac and the two specialized cytosolic proteins p67*^phox^* and p47*^phox^*, each containing two SH3 domains [32], [33]. In this process, p47*^phox^* translocates to the membrane by itself, whereas p67*^phox^* is recruited via p47*^phox^* [34], [35]: they constitutively associate via the interaction of the C-terminal SH3 domain of p67*^phox^* with the p47*^phox^* C-terminus [36], [37]. Thus, p47*^phox^* plays a central role in the membrane translocation. Indeed, our results confirmed that ATPγS-induced COX-2 expression and PGE_2_ synthesis was reduced by pretreatment with a ROS inhibitor (Edaravone) and the inhibitors of NADPH oxidase (DPI or APO) or transfection with p47*^phox^* siRNA. Pretreatment with DPI or APO inhibited ATPγS-induced ROS generation. These results suggested that NADPH oxidase-dependent ROS generation was involved in ATPγS-induced COX-2/PGE_2_ expression. Although the signaling pathways underlying ATPγS-regulated NADPH oxidase have not been completely defined, involvement of PKC in NADPH oxidase activation has been reported in various cell types [15], [38], [39]. This note is confirmed by our observation that ATPγS-induced NADPH oxidase activity, ROS generation, and p47*^phox^* translocation was inhibited by pretreatment with the inhibitors of PKCs.

Among the purinoreceptors, P1Rs (now known as A_1_, A_2_, and A_3_ receptors) respond to adenosine but not to ATP, whereas all P2Rs (P2XR or P2YR) respond to ATP, some also respond to ADP, uridine 5*'*-triphosphate, or uridine 5*'*-diphosphate [5], [26]. In the present study, we found that ATPγS regulated COX-2/PGE_2_ expression, PKC activation, and ROS generation via P2 receptor in A549 cells by pretreatment with the inhibitors of P2 receptors. These data suggested that ATPγS may cause lung and airway inflammation via the P2 receptor-dependent COX-2/PGE_2_ induction.

STATs are a class of transcription factors bearing SH2 domains that become activated upon tyrosine phosphorylation [23], [40]. STAT3 is a transcription factor that is activated by many cytokines and growth factors and plays a key role in cell survival, proliferation, and differentiation [23], [40]. The phosphorylation of STAT3 at Tyr^705^ is most commonly mediated by Jaks, especially Jak2 [17]. COX-2 expession has also been shown to be mediated via STAT3/Jak2 activation [18], [19]. Moreover, this is confirmed by our data that pretreatment with the inhibitor of Jak2 or STAT3 markedly inhibited ATPγS-induced COX-2 expression and PGE_2_ generation in A549 cells. Oxidative stress has been shown to increase the activity of transcription factors, such as STAT3 [40]. Here, we found that NADPH oxidase-dependent ROS production was involved in ATPγS-stimulated Jak2 and STAT3 phosphorylation. Thus, ROS may be critical for the inflammatory responses triggered by ATPγS, through the up-regulation of redox-sensitive transcription factors and hence the expression of proinflammatory genes. Further understanding of the effects and roles of ROS in cellular functions as amplification of proinflammatory and immunological responses, signaling pathways, activation of transcription factors, and gene expression will provide important information regarding pathological processes contributing to chronic lung diseases. In summary, as depicted in Fig. 8, our results showed that ATPγS induced ROS production through a P2 receptor/PKCs/NADPH oxidase signaling, in turn initiated the activation of Jak2 and STAT3. Activated STAT3 was recruited to the promoter region of COX-2 leading to an increase of COX-2 expression associated with PGE_2_ release. Therefore, the inhibitors of P2 receptors may be proven useful in diminishing ATPγS-induced lung inflammation and chronic pathology.

**Figure 8:** Schematic diagram illustrating the proposed signaling pathway involved in ATPγS-induced COX-2 expression and PGE_2_ generation in A549 cells. ATPγS activates the P2 receptor/PKC/NADPH oxidase pathway to enhance ROS generation, which in turn initiates the activation of Jak2 and STAT3, and ultimately induces COX-2-dependent PGE_2_ generation in A549 cells.
